RETRACTED

# Gulf war illness inflammation reduction trial: A phase 2 randomized controlled trial of low-dose prednisone chronotherapy, effects on health-related quality of life

**DOI:** 10.1371/journal.pone.0286817

**Published:** 2023-06-15

**Authors:** Ronald R. Bach, Rebecca R. Rudquist

**Affiliations:** Minneapolis Veterans Affairs Health Care System, Minneapolis, Minnesota, United States of America; Boston University School of Public Health, UNITED STATES

## Abstract

**Background:**

Gulf War illness (GWI) is a deployment-related chronic multisymptom illness impacting the health-related quality of life (HRQOL) of many U.S. Military Veterans of the 1990–91 Gulf War. A proinflammatory blood biomarker fingerprint was discovered in our initial study of GWI. This led to the hypothesis that chronic inflammation is a component of GWI pathophysiology.

**Objectives:**

The GWI inflammation hypothesis was tested in this Phase 2 randomized controlled trial (RCT) by measuring the effects of an anti-inflammatory drug and placebo on the HRQOL of Veterans with GWI. The trial is registered at ClinicalTrials.gov, Identifier: NCT02506192.

**RCT design and methods:**

Gulf War Veterans meeting the Kansas case definition for GWI were randomized to receive either 10 mg modified-release prednisone or matching placebo. The Veterans RAND 36-Item Health Survey was used to assess HRQOL. The primary outcome was a change from baseline in the physical component summary (PCS) score, a measure of physical functioning and symptoms. A PCS increase indicates improved physical HRQOL.

**Results:**

For subjects with a baseline PCS <40, there was a 15.2% increase in the mean PCS score from 32.9±6.0 at baseline to 37.9±9.0 after 8 weeks on modified-release prednisone. Paired t-test analysis determined the change was statistically significant (p = 0.004). Eight weeks after cessation of the treatment, the mean PCS score declined to 32.7±5.8.

**Conclusions:**

The prednisone-associated improvement in physical HRQOL supports the GWI inflammation hypothesis. Determining the efficacy of prednisone as a treatment for GWI will require a Phase 3 RCT.

## Introduction

At least 25% of the 697,000 U.S. military personnel who served in the 1990–91 Gulf War, Operations Desert Shield and Desert Storm, meet a case definition for Gulf War illness (GWI) [1–3]. GWI is a deployment-related chronic multisymptom illness. Symptoms of the syndrome include musculoskeletal pain, chronic fatigue, cognitive impairment, gastrointestinal problems, skin rashes, and respiratory difficulties.

The mission of GWI research is to improve the health-related quality of life (HRQOL) of Veterans with GWI. To this end we have employed a translational research strategy. Our goal was to discover an evidence-based treatment for this deployment-related illness that would alleviate symptoms and mitigate the long-term detrimental health effects of the disorder.

RETRACTED

The process began with the hypothesis that there are biomarkers in blood that will reveal something about the underlying pathophysiology of GWI. To test the hypothesis, we conducted an observational study of blood from Gulf War Veterans who met the Fukuda CDC-10 GWI case definition (GWI+) and those who did not (GWI-) [4]. The blood analysis included peripheral blood counts and plasma proteomics. More than 100 blood parameters were quantified for each subject. Statistical comparison of the GWI+ and GWI- data identified 12 significant blood biomarker differences [5–7].

The biological functions of the 12 GWI-associated biomarkers revealed a proinflammatory biomarker fingerprint. This observation led to the hypothesis that chronic inflammation is an underlying component of GWI pathophysiology. The GWI inflammation hypothesis was tested in a randomized controlled trial (RCT) measuring the effects of an anti-inflammatory drug and placebo on clinically relevant endpoints. The Gulf War Illness Inflammation Reduction Trial (GWIIRT) is a proof-of-concept study. Additional support for the GWI inflammation hypothesis comes from discoveries by other investigators of additional GWI-associated biomarkers of inflammation [8, 9].

The selection of an evidence-based intervention for this study was guided by the identification of a specific therapeutic target. Nuclear factor kappa-light-chain-enhancer of activated B cells (NF-κB) is a transcription factor that functions as a key regulator of inflammation. Activated NF-κB induces the expression of numerous proinflammatory genes including some coding for GWI biomarkers [10, 11]. Therefore, NF-κB was selected as the molecular target for inflammation reduction.

Glucocorticoids (cortisol, cortisone, etc.), have pleiotropic effects on the immune system. Synthetic glucocorticoid derivatives (dexamethasone, prednisone, etc.) are anti-inflammatory drugs that block pro-inflammatory gene expression [12, 13]. Prednisone was selected as the evidence-based intervention for this study because its potent anti-inflammatory activity is mediated, at least in part, by the inhibition of NF-κB activation.

Chronotherapy is the delivery of a medication in coordination with circadian rhythms. The optimal time for delivery of a glucocorticoid is in the early morning hours when the expression of genes coding for proinflammatory cytokines such as IL-6 are at their circadian peaks [14–16]. This evidence led to the development of modified-release (MR) prednisone which is taken at bedtime and programmed for release approximately 4 hours after ingestion. IL-6 is a GWI-associated proinflammatory biomarker [6]. Therefore, chronotherapy was selected as the method of prednisone delivery.

RETRACTED

The efficacy of low-dose prednisone chronotherapy as a treatment for rheumatoid arthritis (RA) has been demonstrated in two Phase 3 RCTs. Circadian Release of Prednisone in Rheumatoid Arthritis (CAPRA)-1 compared MR-prednisone taken at bedtime to the standard immediate-release formulation of prednisone taken in the morning [17]. CAPRA-2 compared MR-prednisone to placebo [18]. Thus, the MR formulation of prednisone was chosen for the GWIIRT.

## Materials and methods

### Study design

The GWIIRT (ClinicalTrials.gov Identifier: NCT02506192) is a Phase 2 randomized, placebo-controlled, double-blind, parallel group, clinical trial. The prednisone arm received a low-dose (10 mg qd) of MR-prednisone for 8 weeks. The placebo arm received matching placebo tablets. The treatment phase was followed by a washout period of 8 weeks. The study goal was to determine if prednisone treatment induces a statistically significant change from baseline in physical HRQOL. Horizon Therapeutics Plc supplied the MR-prednisone (Rayos^®^) and matching placebo for this study at no cost per the Department of Veterans Affairs (VA) Investigator Initiated Clinical Trial Cooperative Research and Development Agreement.

### Eligibility to participate

Inclusion criteria:

- Scores moderately severe or multiple symptoms in at least 3 out of 6 domains from the Kansas GWI Case Definition questionnaire [19]
- Deployed to the Kuwaiti Theater of Operation (August 2, 1990-July 31, 1991) and was honorably discharged

Exclusion criteria:

- Hospitalization anytime since 1990 for alcohol or drug dependence, depression, or PTSD
- Known hypersensitivity to prednisone
- Liver disease, (active or recent Hepatitis B or C treatment with a completion date within the past 6 months, or alcohol liver disease), or kidney disease
- Treated diabetes
- Female who is pregnant or nursing
- Female who refuses to use an accepted method of birth control
- Exclusionary labs: high sensitivity C-reactive protein (hs-CRP) >25 μg/ml, creatinine clearance <30 ml/min, estimated glomerular filtration rate ≤30 ml/min, hemoglobin A1-C >7%, glucose >120 mg/dL, leukocyte count >12x10^6^/ml, erythrocyte count >6.2x10^9^ cells/ml, hematocrit >60%, hemoglobin <11 gm/dL, platelets <10^5^/μL, liver function tests (2 x the upper limit of aspartate aminotransferase and alanine aminotransferase, 2 x the upper limit of total bilirubin and alkaline phosphatase)
- Inflammatory arthritis (RA, psoriatic arthritis, spondylitis, polyarthritis)
- Reactive arthritis, or inflammatory bowel disease-associated arthritis
- Any major inflammatory disease requiring steroid treatment: acute/chronic infections, inflammatory bowel disease, pericarditis, vasculitis, chronic obstructive pulmonary disease, or asthma
- Chronic use of prednisone or other corticosteroids (occasional inhaled use of steroids acceptable)
- Active gum disease or dental infection
- Diagnosed with lupus, stroke, multiple sclerosis (MS), or any other diagnosis that produces symptoms of fatigue, cognitive impairment, or pain
- Any condition that may interfere with the ability to accurately report symptoms (severe psychiatric problems, schizophrenia, bipolar disorder, alcohol, or drug dependence requiring hospitalization, or regular illegal drug use)
- Heart disease (other than hypertension), heart failure or coronary heart disease requiring hospitalization within the past 12 months
- Cancer (other than basal cell skin cancer), requiring treatment within the past 12 months, or life expectancy of less than 1 year
- Hospitalization within the past 3 months

RETRACTED

### Kansas GWI case definition

The Kansas GWI Case Definition questionnaire was administered as a screening tool to determine eligibility to participate in the study. It has both inclusionary and exclusionary components. The Kansas GWI case definition was developed from a population-based survey of over 2,000 Kansas Gulf War Veterans [19]. It is a more comprehensive analysis of eligibility than the Fukuda CDC-10 case definition [4] that was employed in our blood biomarker studies [5–7].

To be considered GWI+ the Veteran must endorse moderately severe or multiple symptoms in at least 3 of 6 symptom domains: fatigue/sleep problems, neurological/cognitive/mood symptoms, pain symptoms, gastrointestinal symptoms, respiratory symptoms, and skin symptoms. In addition, the first appearance of the symptoms must have been either during or after the Gulf War.

### Kansas Symptom Severity (KSS) score

The KSS calculation utilizes the data from the three most prominent symptom domains of the Kansas case definition questionnaire: fatigue/sleep problems, neurological/cognitive/mood symptoms, and pain symptoms. For each survey question, the subjects rated the severity of the symptom. A numerical value was assigned to each symptom severity rating: none = 0, mild = 1, moderate = 2, severe = 3. The scores within each domain were averaged, and the 3 domain averages were summed. Thus, each study subject received a summary score ranging from 0 to 9.

### Primary and secondary outcome measures

The Veterans RAND 36-Item Health Survey (VR-36^©^) was employed as the measure of HRQOL. The VR-36 yields two summary scores: a physical component summary (PCS) and a mental component summary (MCS) [20–24]. For each study subject, the PCS and MCS were determined at baseline (Visit 1), 8 weeks (Visit 2), and 16 weeks (Visit 3). Established methods for calculating these scores were employed [25]. The scores range from 0 (maximum disability) to 100 (no disability). Fifty is the normative value for a particular population. The PCS change from baseline was the primary outcome measure. The MCS change from baseline was the secondary outcome measure.

RETRACTED

### Statistical methods

The PCS and MCS data are presented as the mean score ± standard deviation (std dev). The Shapiro-Wilk test was used to assess normality. The data were normally distributed. Therefore, a paired t-test was employed in the statistical analysis of intragroup changes from baseline at 8 weeks and 16 weeks. The p-values presented are for a two-tailed test. Student’s t-test was used to analyze intergroup changes, e.g., mean values of demographic characteristics for the prednisone and placebo arms of the study. SigmaStat v4.0 statistical software was used for the statistical analyses.

### Recruitment and informed consent

The primary method for recruiting potential subjects was a Minneapolis VA Health Care System (MVAHCS) Investigational Review Board (IRB)-approved recruitment letter sent to Gulf War Veterans listed in the MVAHCS Persian Gulf War Registry. Interested Veterans called the MVAHCS Gulf War Hotline. After the initial medication questions, Veterans answered the Kansas GWI Case Definition questionnaire. In addition to meeting the Kansas criteria, subjects had to be willing to make several trips to the MVAHCS for study visits and to take the study drug or placebo as directed. The recruitment period for this study was from July 1, 2015, to December 31, 2019. The final study visit of the last subject was on April 6, 2020. The process of obtaining informed consent began at the initial appointment and was performed in accordance with good clinical practices guidelines. The GWIIRT protocol, informed consent documents, and waivers for the screening were approved by the MVAHCS IRB.

### Randomization, intent-to-treat, and power analysis

Block randomization was used to assign participants to comparison groups. For each consecutive pair (block) of enrolled subjects, one member was assigned to the treatment arm, the other member to the placebo arm. The pseudo-random number generator in Microsoft Excel was used to generate random numbers to permit the treatment assignment within each block of subjects. Treatment assignment codes were generated and kept by the MVAHCS research pharmacist and stored on a secure VA server behind VA firewalls. All study participants and study personnel, except the research pharmacist, remained blinded to the assignments until the last subject had completed the final study visit.

RETRACTED

An intent-to-treat analysis was used for the outcome measures. All study participants had a calculable PCS and MCS at baseline. Missing values for the two participants who withdrew from the study were set to equal baseline scores (last-observation-carried-forward strategy).

Power analysis was used to establish the GWIIRT recruitment goal. In a VA study of the effects of cognitive behavioral therapy and aerobic exercise on GWI, an intervention-related 7-point increase in the PCS with no change in the placebo arm was defined as clinically significant [26, 27]. Using this value and an estimate of the variability of change, the calculation determined that 40 subjects per group would be needed to detect the difference between medication and placebo of 7 PCS points with 80% power at the p = 0.05 significance level (nQuery Advisor v7).

### Screening and study visit

Following the consenting process, each subject had an IRB-approved screening appointment. The appointment included a physical exam, review of systems, and blood tests. Personal questions, including a list of current medications, were asked on the screening questionnaire. If all eligibility criteria were met, then the VR-36 survey was administered. Subjects answered the questions in a GWI study exam room. Subsequent visits were formatted to provide an experience that was predictable. Consistency of conditions were achieved by using the same appointment time and location as often as possible.

Blood tests performed for screening included a complete blood count (CBC), creatinine, blood glucose, and hemoglobin A1C. The purpose of screening assays was to establish that certain exclusion criteria were not met. Blood tests associated with the study visits evaluated the health of the subjects. The CBC was used to evaluate the possibility of an intercurrent infection. For subject safety blood glucose and hemoglobin A1C were measured at each study visit.

### Treatment

Information regarding the use of the study drug (Instructions for Study Medication) was given to each subject. Subjects were informed of the potential for drug interactions with the study drug. Subjects were instructed to inform their personal physicians that they are participating in a research study involving treatment. The dose of the MR-prednisone employed in this study was 10 mg/qd. At the end of the first study visit each subject received their bottle of 112 tablets, either 5 mg MR-prednisone or matching placebo. The drug and placebo cores were surrounded by a shell matched in appearance for color, size, shape, and embossment. The placebo core contained: 43.8 mg lactose monohydrate, 11 mg croscarmellose sodium, 4 mg providone, 0.3 mg colloidal silicone dioxide, 0.6 mg magnesium stearate, 0.3 mg red ferric oxide. Subjects were instructed to take 2 tablets at bedtime. After 8 weeks each subject returned to the MVAHCS for their second study visit. Bottles were returned to the research pharmacist, and the remaining pills were counted to assess compliance

RETRACTED

## Results

A total of 83 Gulf War Veterans were enrolled in the GWIIRT, Fig 1. Forty-two subjects were randomized to the prednisone arm. Forty-one subjects were randomized to the placebo arm. One subject from each arm withdrew at the second study visit for personal reasons. For the 81 subjects completing the study, based on the number of tablets returned at the second study visit, the compliance rate was 94%.

**Fig 1:** Consort flow diagram.

The demographic characteristics of the Gulf War Veterans enrolled and randomized in the study are presented in Table 1. Student’s t-test was used to determine there were no statistically significant differences in BMI, weight, or age between the two arms of the study. The distributions for all U.S. military personnel deployed in the Gulf War were: 93% male, 7% female, 77% White, 17% Black, and 6% other (Asian, Hispanic, Native American).

**Table 1:** GWIIRT baseline demographic characteristics.

Variable	Total	Placebo	Prednisone
**N**	**83**	**41**	**42**
**BMI, Mean±Std Dev**	**31.6±6.2**	**30.9±6.6**	**32.2±5.8**
**Age (yrs), Mean±Std Dev**	**51.0±5.5**	**49.7±4.0**	**52.2±6.4**
**Weight (lbs), Mean±Std Dev**	**224±46.3**	**222±48**	**228±45**
**Male, N (%)**	**78 (94)**	**38 (94)**	**40 (95)**
**Female, N (%)**	**5 (6.0)**	**3 (7.3)**	**2 (4.8)**
**Race, White, N (%)**	**76 (92)**	**37 (90)**	**39 (93)**
**Black, N (%)**	**4 (4.8)**	**2 (4.9)**	**2 (4.8)**
**Hispanic, N (%)**	**2 (2.4)**	**1 (2.4)**	**1 (2.4)**
**Native American, N (%)**	**1 (1.2)**	**1 (2.4)**	**0 (0)**

To test the validity of the PCS as a measure of changes in GWI symptoms, the hypothetical relationship between the baseline metrics for GWI symptoms severity (KSS) and physical HRQOL (PCS) was evaluated by linear regression analysis, Fig 2. Pearson’s correlation coefficient (r) and the p-value were calculated. The negative linear correlation between KSS and PCS was statistically significant (r = -0.67, p = 7.3E-12).

**Fig 2:** Linear correlation between baseline KSS and baseline PCS.

The primary outcome data, i.e., the change in the mean PCS from baseline (Visit 1) to 8 weeks (Visit 2) and from baseline to 16 weeks (Visit 3), are presented in Table 2. At 8 weeks the mean PCS increased by 2.7 points (6.6%) in the prednisone arm and by 1.9 points (4.2%) in the placebo arm. Both changes were statistically significant. At 16 weeks the mean PCS in each arm returned to baseline. During the washout there were no reports of adverse reactions related to the cessation of either drug or placebo.

RETRACTED

**Table 2:** PCS changes from baseline in the prednisone and placebo arms.

Study Arm	Visit #	N	PCS Mean	Std Dev	ΔPCS V1→V2	P Value*	ΔPCS V1→ V3	P Value*
**Prednisone**	**1**	**42**	**40.8**	**±9.2**				
	**2**		**43.5**	**±9.6**	**2.7**	**0.009**		
	**3**		**40.8**	**±8.3**			**0**	**0.97**
**Placebo**	**1**	**41**	**41.5**	**±9.9**				
	**2**		**43.4**	**±9.8**	**1.9**	**0.046**		
	**3**		**41.4**	**±10.8**			**-0.1**	**0.96**

*Paired t-test

Subgroup analysis was employed to evaluate the possibility of a correlation between the PCS levels at baseline and the primary outcome results. Each arm of the study was divided into two subgroups based on the baseline scores. Study subjects were identified as either low PCS (baseline PCS <40) or high PCS (baseline PCS >40). The dividing line of 40 points was chosen a priori for an equitable distribution of subjects. Results of the subgroup analysis are presented in Table 3.

**Table 3:** Subgroup analysis of PCS changes from baseline.

Study Arm	Visit #	Baseline PCS	N	PCS Mean*	Std Dev	ΔPCS V1→V2	P Value	ΔPCS V1→ V3	P Value
**Prednisone**	**1**	**Low**	**19**	**32.9**	**±6.0**				
	**2**			**37.9**	**±9.0**	**5.0**	**0.004**		
	**3**			**32.7**	**±5.8**			**-0.2**	**0.77**
**Placebo**	**1**	**Low**	**20**	**32.9**	**±4.5**				
	**2**			**35.9**	**±6.4**	**3.0**	**0.043**		
	**3**			**33.8**	**±6.5**			**0.9**	**0.39**
**Prednisone**	**1**	**High**	**23**	**47.3**	**±5.5**				
	**2**			**48.1**	**±7.5**	**0.8**	**0.49**		
	**3**			**47.5**	**±6.8**			**0.2**	**0.88**
**Placebo**	**1**	**High**	**21**	**49.6**	**±5.7**				
	**2**			**50.6**	**±6.5**	**1.0**	**0.47**		
	**3**			**48.7**	**±9.0**			**-0.9**	**0.55**

*Paired t-test

In the low PCS prednisone subgroup, there was a statistically significant increase of 5.0 points (15.2%) in the mean PCS at 8 weeks, p = 0.004. In the low PCS placebo subgroup, there was a statistically significant increase of 3.0 points (9.1%) in the mean PCS at 8 weeks, p = 0.043. After the washout, the mean scores in both low PCS subgroups returned to baseline levels. No statistically significant change in the mean PCS of either high PCS subgroup was observed.

The MCS data are presented in Table 4. In the prednisone arm there was a mean MCS increase of 1.6 points at 8 weeks that was not statistically significant, p = 0.14. In the placebo arm there was a mean MCS increase of 2.7 points at 8 weeks that was statistically significant, p = 0.023. The mean MCS in the prednisone arm returned to baseline at 16 weeks. The mean MCS in the placebo arm remained elevated at 16 weeks but lost statistical significance.

RETRACTED

**Table 4:** MCS changes from baseline in the prednisone and placebo arms.

Study Arm	Visit #	N	MCS Mean	Std Dev	ΔMCS V1→V2	P Value*	ΔMCS V1→ V3	P Value*
**Prednisone**	**1**	**42**	**40.8**	**±13.3**				
	**2**		**42.4**	**±13.2**	**1.6**	**0.14**		
	**3**		**40.1**	**±12.4**			**-0.7**	**0.59**
**Placebo**	**1**	**41**	**40.4**	**±12.8**				
	**2**		**43.1**	**±11.9**	**2.7**	**0.023**		
	**3**		**42.7**	**±12.0**			**2.3**	**0.12**

*Paired t-test

The MCS subgroup data are presented in Table 5. For the low PCS subgroups, there were no statistically significant changes in the mean MCS from baseline. For the high PCS subgroups, the mean MCS increase at 8 weeks was statistically significant for both the prednisone subgroup, p = 0.015, and the placebo subgroup, p = 0.021. At 16 weeks, the mean MCS of the high PCS prednisone subgroup approached the baseline level, while the mean MCS of the high PCS placebo subgroup remained elevated but lost statistical significance.

**Table 5:** Subgroup analysis of MCS changes from baseline.

Study Arm	Visit #	Baseline PCS	N	MCS Mean	Std Dev	ΔMCS V1→V2	P Value*	ΔMCS V1→ V3	P Value*
**Prednisone**	**1**	**Low**	**19**	**35.6**	**±12.4**				
	**2**			**35.1**	**±11.4**	**-0.5**	**0.75**		
	**3**			**33.0**	**±8.7**			**-2.6**	**0.29**
**Placebo**	**1**	**Low**	**20**	**39.1**	**±11.4**				
	**2**			**40.0**	**±12.1**	**0.9**	**0.49**		
	**3**			**39.1**	**±11.7**			**0**	**0.96**
**Prednisone**	**1**	**High**	**23**	**45.1**	**±12.8**				
	**2**			**48.3**	**±11.6**	**3.2**	**0.015**		
	**3**			**46.0**	**±12.0**			**0.9**	**0.44**
**Placebo**	**1**	**High**	**21**	**41.7**	**±14.1**				
	**2**			**45.9**	**±11.3**	**4.2**	**0.021**		
	**3**			**46.0**	**±11.6**			**4.3**	**0.09**

*Paired t-test

## Discussion

Employing the change in physical HRQOL from baseline as the primary outcome measure for this study assumes that a prednisone-induced decrease in GWI symptoms, i.e., reduced KSS, will translate into improved physical HRQOL, i.e., increased PCS. The statistically significant negative linear correlation between KSS and PCS, Fig 2, supports the choice of physical HRQOL as the primary outcome measure.

The potential relevance of the observed prednisone-related increase in the PCS to the long-term health and well-being of GWI+ Veterans was evaluated by comparing the results of CAPRA-2 and the GWIIRT. Both studies were placebo-controlled RCTs employing low-dose prednisone chronotherapy as the intervention. For CAPRA-2, the mean PCS changes from baseline at 12 weeks were 3.6^prednisone^ and 1.3^placebo^. For the GWIIRT low PCS subgroups, the mean PCS changes from baseline at 8 weeks were 5.0^prednisone^ and 3.0^placebo^. Thus, the PCS increases attributable to prednisone were 2.3 points in CAPRA-2 and 2.0 points in the GWIIRT. The near equivalence of the PCS responses to MR-prednisone in the two studies is encouraging. However, RA and GWI are very different disorders. Proving the efficacy of low-dose prednisone chronotherapy as a treatment for GWI will require a Phase 3 RCT.

RETRACTED

Many RA clinical trials have reported robust placebo effects [28]. Significant placebo-related changes in objective markers of inflammation and subjective pain ratings have been observed [29, 30]. Whether the placebo effect on PCS observed in this study is in any way related to the placebo effect observed in RA clinical trials remains to be determined. Analyses of GWIIRT secondary outcome data for placebo-related changes in objective blood biomarkers of inflammation and subjective pain perception may shed light on this question.

Power analysis was used to estimate the minimum sample size of a prospective Phase 3 RCT. Using the low PCS subgroup mean PCS values at 8 weeks and the weighted mean std dev (σ = 7.67), the calculation determined that at least 231 subjects per group would be needed to detect a 2-point difference in the PCS between prednisone and placebo with 80% power at the p = 0.05 significance level. Thus, with the addition of baseline PCS <40 to the inclusion criteria, a Phase 3 RCT of low-dose prednisone chronotherapy is feasible.

All statistically significant PCS changes occurred in the low PCS subgroups. All statistically significant MCS changes occurred in the high PCS subgroups. These divergent subgroup responses indicate there are substantial pathophysiologic differences between the two ends of the PCS spectrum in GWI.

Inflammatory diseases, e.g., RA, multiple sclerosis, and inflammatory bowel disease, can fluctuate between periods of active disease which respond to prednisone treatment and periods of remission which are unresponsive. The evidence in this study that the low PCS subgroup responded to prednisone with improved physical HRQOL, and the high PCS subgroup did not, is consistent with the hypothesis that GWI is a relapsing-remitting inflammatory illness.

The treat-to-target strategy is a widely accepted management paradigm for relapsing-remitting inflammatory diseases. First, an anti-inflammatory drug is used to treat active disease. Management goals are evaluated by regular assessments of disease activity using objective outcome measures. If remission is achieved, then sustaining the remission becomes the new objective [31–36]. A treat-to-target strategy should be considered for the long-term care of GWI+ Veterans.

RETRACTED

The prednisone-induced PCS increase returned to the baseline level following cessation of treatment. In this Phase 2 study there was only one treatment time point at 8 weeks. The effects of longer treatment are unknown. It is possible that continuation of low-dose prednisone chronotherapy will result in higher PCS levels and maintaining the maximum prednisone effect may produce a stable steady state that is no longer drug dependent, i.e., remission [37]. This GWI remission hypothesis is testable.

The inflammaging hypothesis proposes that chronic inflammation accelerates the normal aging process [38, 39]. Also, chronic inflammation contributes significantly to the morbidity and mortality of age-related diseases, e.g., atherosclerosis, cardiovascular disease, cancer, type-2 diabetes, hypertension, and Alzheimer’s disease. [40, 41]. Therefore, reducing chronic inflammation in GWI+ Veterans, in addition to increasing physical HRQOL, may have other long-term health benefits.

Unexplained illnesses have been reported by many U.S Military Veterans of more recent deployments to Iraq and Afghanistan. Burn pits are one source of toxic exposures that may be responsible for this emerging pathophysiology. The burn pit syndrome manifests GWI-like symptoms [42]. Thus, the translational research strategy employed in this study of GWI may be a productive path for investigations of this new wave of deployment-related illness.

### Strengths

The hypothesis that chronic inflammation is a component of GWI pathophysiology was based on objective blood biomarker evidence. Likewise, the choice of low-dose prednisone chronotherapy as the intervention was evidence-based. The RCT study design is strong. The results of this Phase 2 RCT establish the feasibility of a Phase 3 RCT.

### Limitations

This is a small Phase 2 RCT, and the results have not been replicated. A Phase 3 RCT is required to demonstrate efficacy and obtain regulatory approval of low-dose prednisone chronotherapy as a treatment for GWI.

## Conclusions

After 8 weeks of low-dose prednisone chronotherapy, there was a statistically significant increase in the physical HRQOL of GWI+ Veterans with baseline PCS <40. This result supports the hypothesis that chronic inflammation is a component of GWI pathophysiology. A Phase 3 RCT is necessary to determine the efficacy of low-dose prednisone chronotherapy as a treatment for GWI.

RETRACTED

## Supporting information

S1 Checklist CONSORT 2010 checklist of information to include when reporting a randomised trial*. (DOC)

S1 Data (XLSX)

S1 File Gulf war illness inflammation reduction trial protocol: September 12, 2013. (DOCX)

S2 File (DOCX)

## References

[1] Research Advisory Committee on Gulf War Veterans’ Illnesses. Gulf War Illness and the Health of Gulf War Veterans: Scientific Findings and Recommendations. Washington, D.C.: U.S. Government Printing Office, 2008.

[2] Institute of Medicine of the National Academies Committee on Gulf War and Health. Gulf War and Health, Volume 8: Update of Health Effects of Serving in the Gulf War. Washington, DC: The National Academies Press. 2009.

[3] WhiteRF, SteeleL, O’CallaghanJP, et al: Recent research on Gulf War illness and other health problems in veterans of the 1991 Gulf War: Effects of toxicant exposures during deployment. Cortex. 2016; 74: 449–475. doi: 10.1016/j.cortex.2015.08.022 26493934PMC4724528

[4] FukudaK, NisenbaumR, StewartG, et al: Chronic multisymptom illness affecting Air Force veterans of the Gulf War. JAMA. 1998;280(11):981–988. doi: 10.1001/jama.280.11.981 9749480

[5] JohnsonGJ, SlaterBC, LeisLA, RectorTS, BachRR: Blood Biomarkers of Chronic Inflammation in Gulf War Illness. PLOS ONE. 2016 Jun 28;11(6). doi: 10.1371/journal.pone.0157855 27352030PMC4924830

[6] ButterickTA, TrembleyJH, Hocum StoneLL, MullerCJ, RudquistRR, BachRR: Gulf War Illness-associated increases in blood levels of interleukin 6 and C-reactive protein: biomarker evidence of inflammation. BMC Res Notes. 2019; 12: 816. doi: 10.1186/s13104-019-4855-2 31852524PMC6921550

[7] JohnsonGJ, LeisLA, SlaterBC, BachRR: Elevated platelet count, C-reactive protein, and thromboxane analog-induced platelet aggregation in patients with Gulf War Veterans’ illnesses: evidence of a chronic inflammatory state? Blood coagulation & fibrinolysis: an international journal in haemostasis and thrombosis. 2013;24(7):736–41. doi: 10.1097/MBC.0b013e328362627f 23751609

[8] KhaiboullinaSF, DeMeirleirKL, RawatS, et al. Cytokine expression provides clues to the pathophysiology of Gulf War illness and myalgic encephalomyelitis. *Cytokine*. 2015;72(1):1–8. doi: 10.1016/j.cyto.2014.11.019 25514671PMC4410698

[9] JanulewiczPA, SethRK, CarlsonJM, et al. The Gut-Microbiome in Gulf War Veterans: Preliminary Report. *Int J Environ Res Public Health*. 2019;16(19): 3751.3159032210.3390/ijerph16193751PMC6801913

[10] GilmoreTD: Introduction to NF-κB: players, pathways, perspectives. Oncogene. 2006;2: 6680–6684.10.1038/sj.onc.120995417072321

[11] LiuT, ZhangL, JooD, SunSC: NF-κB signaling in inflammation. Signal Transduction and Targeted Therapy. 2017;2: Article ID 17023.10.1038/sigtrans.2017.23PMC566163329158945

RETRACTED

[12] HardyRS, RazaK, CooperMS: Therapeutic glucocorticoids: mechanisms of actions in rheumatic diseases. Nat Rev Rheumatol. 2020;16, 133–144. doi: 10.1038/s41584-020-0371-y 32034322

[13] CainD, CidlowskiJ: Immune regulation by glucocorticoids. Nat Rev Immunol. 2017;17, 233–247. doi: 10.1038/nri.2017.1 28192415PMC9761406

[14] SelfridgeJM, GotohT, SchiffhauerS, et al: Chronotherapy: Intuitive, Sound, Founded…But Not Broadly Applied. Drugs. 2016; 76(16): 1507–1521.2769964410.1007/s40265-016-0646-4PMC5082589

[15] Glass‐MarmorL, PapernaT, Ben‐YosefY, MillerA: Chronotherapy using corticosteroids for multiple sclerosis relapses. J Neurol Nurosurg Psychiatry. 2007; 78(8): 886–888. doi: 10.1136/jnnp.2006.104000 17056624PMC2117717

[16] KirwanJ: Targeting the time of day for glucocorticoid delivery in rheumatoid arthritis. Int J Clin Rheum. 2011; 6: 273–279.

[17] ButtgereitF, DoeringG, SchaefflerA, et al: Efficacy of modified-release versus standard prednisone to reduce duration of morning stiffness of the joints in rheumatoid arthritis (CAPRA-1): a double-blind, randomized controlled trial. Lancet. 2008; 371: 205–14.1820701610.1016/S0140-6736(08)60132-4

[18] ButtgereitF, MehtaD, KirwanJ: Low-dose prednisone chronotherapy for rheumatoid arthritis: a randomized clinical trial (CAPRA-2). Ann Rheum Dis. 2013; 72(2):204–210.2256297410.1136/annrheumdis-2011-201067PMC3553491

[19] SteeleL: Prevalence and patterns of Gulf War illness in Kansas veterans: association of symptoms with characteristics of person, place, and time of military service. Am J Epidemiol. 2000;152(10):992–1002. doi: 10.1093/aje/152.10.992 11092441

[20] Kazis LE, Skinner K, Rogers W, Lee A, Ren XS, Miller D: Health Status and Outcomes of Veterans: Physical and Mental Component Summary Scores (SF-36V). Washington, DC, and Bedford, Mass: Office of Performance and Quality, Health Assessment Project, Center for Health Quality Outcomes and Economic Research, HSR&D Service, and Veterans Administration; July 1998.

[21] KazisLE, MillerDR, ClarkJ, et al: Health related quality of life in patients served by the Department of Veterans Affairs: results from the Veterans Health Study. Archives of Internal Medicine. 1998; 158(6): 626–632. doi: 10.1001/archinte.158.6.626 9521227

[22] KazisLE, RenXS, LeeA, et al: Health status in VA patients: results from the Veterans Health Study using the Veterans SF-36. American Journal of Medical Quality. 1999; 14(1): 28–38.1044666110.1177/106286069901400105

[23] KazisLE, MillerDR, ClarkJ, et al: Improving the response choices on the veterans SF-36 health survey role functioning scales: results from the Veterans Health Study. J Ambul Care Manage. 2004; 27(3): 264–280. doi: 10.1097/00004479-200407000-00010 15287216

RETRACTED

[24] KazisLE, SelimA, RogersW, et al: Dissemination of methods and results from the veterans health study: final comments and implications for future monitoring strategies within and outside the veterans healthcare system. J Ambul Care Manage. 2006; 29(4): 310–319. doi: 10.1097/00004479-200610000-00007 16985389

[25] TaftC, KarlssonJ, SullivanM: Do SF-36 summary component scores accurately summarize subscale scores? Qual Life Res. 2001; 10(5): 395–404. doi: 10.1023/a:1012552211996 11763202

[26] DontaST, ClauwDJ, EngelCC, et al: Cognitive behavioral therapy and aerobic exercise for Gulf War veterans’ illnesses: A randomized controlled trial. JAMA. 2003; 289: 1396–1404. doi: 10.1001/jama.289.11.1396 12636462

[27] GuarinoP, PeduzziP, DontaST, et al: A multicenter two by two factorial trial of cognitive behavioral therapy and aerobic exercise for Gulf War veterans’ illnesses: Design of a Veterans Affairs Cooperative Study (CSP #470). Controlled Clinical Trials. 2001; 22: 310–332. doi: 10.1016/s0197-2456(00)00133-1 11384792

[28] BechmanK, YatesM, NortonS, et. al. Placebo Response in Rheumatoid Arthritis Clinical Trials. J Rheumatol. 2020; 47(1): 28–34. doi: 10.3899/jrheum.190008 31043548PMC6941937

[29] VollertJ, CookNR, Kaptcjuk, et al. Assessment of Placebo Response in Objective and Subjective Outcome Measures in Rheumatoid Arthritis Clinical Trials. JAMA Netw Open. 2020;3(9): e2013196. doi: 10.1001/jamanetworkopen.2020.13196 32936297PMC7495232

[30] CollocaL. The Placebo Effect in Pain Therapies. Annu Rev Pharmacol Toxicol. 2019; 59: 191–211. doi: 10.1146/annurev-pharmtox-010818-021542 30216744PMC6402571

[31] AletahaD, WardMM, et al: Remission and active disease in rheumatoid arthritis: defining criteria for disease activity states. Ather Rheum. 2005; 52(9):2625–2636. doi: 10.1002/art.21235 16142705

[32] BacalaoEJ, GreeneGJ, BeaumontJL, et al: Standardizing and personalizing the treat to target (T2T) approach for rheumatoid arthritis using the Patient-Reported Outcomes Measurement Information System (PROMIS): baseline findings on patient-centered treatment priorities. Clin Rheumatol. 2017; 36(8): 1729–1736. doi: 10.1007/s10067-017-3731-5 28653263

[33] SmithAL, CohenJA, HuaLH: Therapeutic Targets for Multiple Sclerosis: Current Treatment Goals and Future Directions. Neurotherapeutics. 2017; 14(4): 952–960. doi: 10.1007/s13311-017-0548-5 28653282PMC5722758

[34] AgrawalM, ColombelJ-F: Treat-to-Target in Inflammatory Bowel Diseases, What Is the Target and How Do We Treat? Gastrointest Endosc Clin N Am. 2019; 29(3): 421–436. doi: 10.1016/j.giec.2019.02.004 31078245

RETRACTED

[35] BurriE, MaillardM, SchoepferAM, et al: Treatment Algorithm for Mild and Moderate-to-Severe Ulcerative Colitis: An Update. Digestion 2020; 101(suppl 1): 2–15 doi: 10.1159/000504092 31945767

[36] SinghJA, SaagKG, BridgesL, et al: 2015 American College of Rheumatology Guideline for the Treatment of Rheumatoid Arthritis. Arthritis Care and Research. 2016; 68(1): 1–25. doi: 10.1002/acr.22783 26545825

[37] FranceschiC, BonafèM, ValensinS, et al: Inflamm-aging. An evolutionary perspective on immunosenescence. Ann N Y Acad Sci. 2000; 908:244–254. doi: 10.1111/j.1749-6632.2000.tb06651.x 10911963

[38] AjeganovaS, HuizingaT. Sustained remission in rheumatoid arthritis: latest evidence and clinical considerations. Ther Adv Musculoskelet Dis. 2017; 9(10): 249–262. doi: 10.1177/1759720X17720366 28974987PMC5613855

[39] SanadaF, TaniyamaY, MuratsuJ, et al: Source of Chronic Inflammation in Aging. Front Cardiovasc Med. 2018; 5:12. doi: 10.3389/fcvm.2018.00012 29564335PMC5850851

[40] ChungHY, KimDH, LeeEK, et al: Redefining Chronic Inflammation in Aging and Age-Related Diseases: Proposal of the senoinflammation concept. Aging and disease. 2019; 10(2):367–382. doi: 10.14336/AD.2018.0324 31011483PMC6457053

[41] WoodsJ, WilundKR, MartinSA, KistlerBM: Exercise, inflammation, and aging. Aging Dis. 2012;3(1):130–140. 22500274PMC3320801

[42] McAndrewsLM, HelmerDA, et al: Iraq and Afghanistan Veterans report symptoms consistent with chronic multisymptom illness on year after deployment. J Rehabil Res Dev. 2016; 53(1): 59–70.2700617310.1682/JRRD.2014.10.0255

